# Long Noncoding RNAs: New Regulators of Resistance to Systemic Therapies for Gastric Cancer

**DOI:** 10.1155/2021/8853269

**Published:** 2021-01-06

**Authors:** Weihong Sun, Changqing Jiang, Ying Ji, Chao Xiao, Haiping Song

**Affiliations:** ^1^Department of Internal Medicine-Oncology Affiliated Qingdao Central Hospital, Qingdao University, 127 Siliu South Road, Qingdao 266042, China; ^2^Department of Internal Medicine-Oncology Qingdao Tumor Hospital, 127 Siliu South Road, Qingdao 266042, China; ^3^Department of Pathology Qingdao Municipal Hospital, Donghai Middle Road, Qingdao 266071, China

## Abstract

Gastric cancer (GC) is the second leading cause of cancer mortality and the fourth most commonly diagnosed malignant disease, with approximately 951,000 new cases diagnosed and approximately 723,000 cases of mortality each year. The highest mortality rate of GC is in East Asia, and the lowest is in North America. A large number of studies have demonstrated that GC patients are characterized by higher morbidity, metastasis rates, and mortality and lower early diagnosis rates, radical resection rates, and 5-year survival rates. All cases of GC can be divided into two important stages, namely, early- and advanced-stage GC, and the stage mainly determines the treatment strategy for and the therapeutic effect in GC patients. Patients with early-stage GC undergo radical surgery followed by chemotherapy, and the 5-year survival rate can be as high as 90%. However, patients with advanced-stage GC cannot undergo radical surgery because they are at risk for metastasis; therefore, they can choose only radiotherapy or chemotherapy and have a poor prognosis. Based on the lack of specific clinical manifestations and detection methods, most GC patients (>70%) are diagnosed in the advanced stage; therefore, continued efforts toward developing treatments have been focused on advanced-stage GC patients and include molecular targeted therapy, immunotherapy, and small molecular therapy. Nevertheless, in recent years, accumulating evidence has indicated that small molecules, especially long noncoding RNAs (lncRNAs), are involved in the occurrence, development, and progression of GC, and their abundantly dysregulated expression has been identified in GC tissues and cell lines. Therefore, lncRNAs are considered easily detectable molecules and ideal biomarkers or target-specific agents for the future diagnosis or treatment of GC. In this review, we primarily discuss the status of GC, the role of lncRNAs in GC, and the emerging systemic treatments for GC.

## 1. Background

### 1.1. Gastric Cancer (GC)

GC continues to be the fourth most common gastrointestinal malignancy, and epidemiological surveys have clearly reported that there are more than 951,000 new cases of GC diagnosed per year and more than 723,000 deaths attributed to it, making GC the third leading cause of cancer-related death worldwide, following lung cancer and liver cancer [1, 2]. Therefore, GC is undoubtedly a serious threat to the health of patients. According to Lauren's criterion, which is the most widely accepted method for GC histologic classification, GC is divided into 4 major subtypes: intestinal, diffuse, mixed, and unclassified [3, 4]. The main differences between intestinal-type GC and diffuse-type GC are that intestinal-type GC is usually exophytic, ulcerating, and often located in the proximal stomach, while diffuse-type GC indicates a poor prognosis and is predominately found in younger patients [5]. Accumulating evidence has demonstrated that many risk factors are implicated in the carcinogenesis and progression of GC, such as genetic factors, obesity, *Helicobacter pylori* infection, Epstein-Barr virus infection, unhealthy diet (for example, high intake of salt and nitrates), hypoxic stress, smoking, pernicious anemia, and chronic atrophic gastritis [1, 6, 7]. Moreover, the occurrence of GC varies with geographic area, with more than 50% of new GC cases and deaths occurring in East Asia, especially in China and Japan [8, 9]. Additionally, it has been found that the incidence of GC is twice as high in men than in women, implying that hormonal differences may also be risk factors for GC progression [10, 11]. In recent years, with the development of enteroscopy and surgical techniques, the five-year overall survival rate for early-stage GC patients has significantly improved, but for advanced-stage GC patients, the five-year survival rate is still unsatisfactory at <25% [12, 13]. The high mortality of GC is mainly attributed to delayed diagnosis due to the absence of screening programs; the lack of desirable molecular biomarkers and the paucity of specific early clinical symptoms; and the common forms of recurrence, including peritoneal dissemination, hematogenous spread, and lymph node metastasis [14, 15]. Thus, patients diagnosed with GC at an advanced stage have missed the best opportunity for curative surgery, and these studies have specifically emphasized the urgent need to seek new biomarkers for the early diagnosis of GC and in-depth investigations into the molecular basis of GC, which is expected to offer novel insights into GC pathogenesis and to further the development of more effective, less toxic, and individualized treatment strategies in the future.

### 1.2. Long Noncoding RNAs (lncRNAs)

A lncRNA is simply defined as a transcript that has an obvious lack of open reading frames (ORFs), has no capacity for coding proteins, and is more than 200 nucleotides (nt) in length. lncRNAs are able to regulate gene expression at various levels, including at the epigenetic, transcriptional, posttranscriptional levels, and are involved in various pathophysiological processes, such as genetic imprinting, cell-directed differentiation, cell proliferation, the cell cycle, tumorigenesis, development of neurodegenerative diseases, development and differentiation of immune cells, and regulation of immune response [16, 17]. Based on their genomic localization and orientation according to their neighboring protein-coding gene, lncRNAs are mainly classified into five types (Figure 1(a)): intergenic lncRNAs (also termed large intervening ncRNAs or lncRNAs, in which the entire lncRNA sequence, as a distinct unit, is located between two protein-coding genes); intronic lncRNAs (the entire lncRNA sequence is located within the intron of a protein-coding gene); bidirectional lncRNAs (the lncRNA expression and that of the neighboring protein-coding genes on the opposite strand are initiated when in close genomic proximity); sense lncRNAs (lncRNA is initiated inside the 5′ end of a protein-coding gene, then transcribed in the same direction as the protein-coding genes, overlapping with at least one protein-coding exon); and antisense lncRNAs (lncRNA is initiated inside the 3′ end of a protein-coding gene and then transcribed in the opposite direction of the protein-coding genes, overlapping with at least one protein-coding exon) [18, 19]. In fact, although lncRNAs have no apparent coding capacity, most of them can be transcribed by the RNA polymerase II (Pol II) complex from any location throughout the genome, and a small portion is synthesized by the RNA polymerase III (Pol III) complex or the single-polypeptide nuclear RNA polymerase IV (spRNAP IV) complex. Subsequently, similar to protein-coding RNAs, transcribed lncRNA transcripts undergo 5′-capping, in a multiexonic structure, 3′-polyadenylation, alternative splicing modifications, and RNA editing procedures through the complete lncRNA transcriptional process. Eventually, lncRNAs are released and transported to subcellular structure locations (e.g., nucleus, nucleolus, cytoplasm, or mitochondria) according to their functions [20, 21].

In the past several years, numerous publications have unequivocally revealed that the manner in which lncRNAs function is diverse, including their involvement in epigenetic regulation by modifying chromatin complexes at specific chromatin sites, regulation of gene transcription by recruitment of transcription factors (TFs), posttranscriptional regulation by selective splicing or the recruitment of RNA to nuclear regions, and regulation of protein translation by acting on protein translation complexes [22, 23]. Regardless of which function a lncRNA exerts, it has been concluded that lncRNAs can function as four regulatory molecules, namely, a signal molecule, a decoy molecule, a guide molecule, and a scaffold molecule (Figure 1(b)) [24, 25]. Nevertheless, no studies have shown that a lncRNA represents only one of these functions; therefore, lncRNAs might function through the integrated manifestation of all the functions described above [26]. First, lncRNAs serve as signal molecules that can integrate developmental cues, interpret cell status or respond to multiple stimuli, and further regulate the expression of other genes in a specific time and space [27]. Second, lncRNAs act as decoy molecules that can associate with DNA-binding proteins to prevent their binding to DNA recognition elements [28]. Third, lncRNAs function as guide molecules that can combine with protein complexes, such as chromatin modification enzymes, to form lncRNA-protein complexes that impart specificity at proper genomic locations [27, 29]. Finally, lncRNAs are considered scaffold molecules that are equivalent to adaptors or assembly platforms that bring two or more proteins into discrete complexes and ultimately change the expression of these genes and their related genes [28, 30]. Hence, based on their multifunctional regulatory mechanisms, lncRNAs comprise a novel field of study that has gained attention and is attractive to the scientific community investigating the occurrence and development processes of human diseases, such as cardiovascular syndromes, diabetes, autoimmune diseases, nervous system disorders, and cancers [31, 32].

### 1.3. lncRNAs and GC

Previous studies have hypothesized that GC is a genetic disease involving multistep changes in the genome; therefore, pervasive studies over the past decades have mostly focused on the interactions between protein-coding genes and GC [33, 34]. Nevertheless, the human genome sequencing project has definitively uncovered that, in the whole human genome, less than 2% of the genome has protein-coding genes (nearly 20,000), whereas almost 98% of the genome is dynamically, pervasively, and actively transcribed into noncoding RNAs (ncRNAs), which were formerly regarded as transcriptional “noise” or body “garbage” [35, 36]. Generally, ncRNAs are classified as lncRNAs (longer than 200 nt) and small ncRNAs (shorter than 200 nt and include microRNAs (miRNAs), small interfering RNAs (siRNAs), Piwi-interacting RNAs (piRNAs), ribosomal RNAs (rRNAs), transfer RNAs (tRNAs), small nuclear RNAs (snRNAs), and small nucleolar RNAs (snoRNAs)) [37]. In the last few decades, numerous studies have convincingly shown that ncRNAs participate in controlling every level of gene expression in diverse cellular processes, such as cell proliferation, growth, apoptosis, migration, and invasion, and in addition, the dysregulated expression of ncRNAs greatly contributes to the initiation, progression, and metastasis of cancers [38, 39]. Therefore, ncRNAs are considered promising biomarker candidates for cancer detection, and the epigenetic mechanisms of ncRNAs that govern GC have also been at the center of GC research in recent years [40, 41].

In recent decades, miRNAs have moved to the forefront of ncRNA research in GC [42, 43]. For instance, miR-345 inhibits the proliferation, migration, and epithelial-mesenchymal transition (EMT) of GC cells by targeting forkhead box Q1 (FoxQ1) [44]; miR-127 curbs GC cell migration and invasion by targeting Wnt7a [45]; miR-1265 suppresses GC progression and oncogenic autophagy by inhibiting calcium-binding protein 39 (CAB39) expression and regulating the AMPK-mTOR signaling pathway [46]; miR-17, miR-25, and miR-133b in circulating serum could be introduced as potential diagnostic candidates applicable for use with early-stage GC patients [47]. However, lncRNAs in GC tumorigenesis are emerging as new players, as has been demonstrated by increasing evidence (illustrated in Table 1) [48, 49]. Furthermore, with the rapid advances in experimental and computational technologies, several hundred aberrantly expressed lncRNAs have been discovered in GC, and their detailed functions have also been revealed [50, 51]. For example, long noncoding small nucleolar RNA host gene 7 (lncRNA SNHG7) is upregulated in GC tissues and cells, and its abnormal expression might play a contributing role in promoting the proliferation and in inhibiting the apoptosis of GC cells by regulating p15 and p16 expression [52]. Long noncoding maternally expressed gene 3 (lncRNA MEG3) is highly expressed in tissues adjacent to corresponding GC tissues, where it is not as highly expressed, and its overexpression could impede the proliferation and metastasis of GC cells by mediating the p53 signaling pathway [53]. In addition, it was found that lncRNAs could act as competing endogenous RNAs (ceRNAs) by sponging miRNAs and are further involved in the indirect regulation of miRNA targets [54]. For instance, lncRNA SLC25A5-AS1/miR-19a-3p/PTEN works as a ceRNA system to facilitate cell growth and inhibit the apoptosis of GC cells [55]. The upregulated lncRNA zinc finger E-box-binding homeobox 2 antisense RNA 1 (ZEB2-AS1) accelerates cell proliferation and metastasis through the miR-143-5p/HIF-1*α* axis [56]. Hence, GC-related lncRNAs serve as potential diagnostic markers and therapeutic targets in clinical applications [57].

## 2. Treatment Strategies for GC

GC remains one of the most frequently occurring and common malignant tumors in the world, with almost 1,000,000 new cases diagnosed each year [6, 58]. In China, the morbidity and mortality of GC are second only to those of lung cancer [10]. At present, the main treatments for GC patients include surgery, chemotherapy, and radiotherapy [9]. Although radical surgery may cure early-stage GC patients, based on the advances in diagnostic strategies with a highly prognostic effect, most patients are already in an advanced stage at the time of treatment due to the hidden nature of the initial symptoms of GC [13, 58]. For patients with advanced-stage GC, radical surgery does not give satisfactory results, and although the administration of chemotherapy drugs can prolong survival and improve quality of life, it also produces many side effects, and high drug resistance leads to a poor prognosis [59, 60]. With the development of medical immunology and molecular biology technology, molecular targeted therapy, immunotherapy, and small molecular therapy have received extensive attention in the field of cancer treatment as an emerging treatment [61, 62]. Therefore, we further explored the progress of these emerging treatments in the clinical study of GC.

### 2.1. Molecular Targeted Therapy

In recent years, molecular targeted therapy has become a focus and hot spot in the field of cancer treatment, and advantages such as low toxicity and high efficiency in the treatment of non-small-cell lung cancer, breast cancer, gastrointestinal stromal tumor, and colorectal cancer have been shown [63]. At this stage, the greatest research progress has been made in the field of molecular targeted therapy for GC [64]. These areas mainly concern epidermal growth factor receptor (EGFR) family-targeting agents, antiangiogenesis, and so on [65, 66]. The roles of lncRNAs in gastric cancer therapy have been reported (Figure 2).

#### 2.1.1. EGFR Family-Targeting Agents

Uncontrolled tumor cell proliferation is one of the prerequisites for cancer to progress rapidly [38]. The EGFR family, also termed the ErbB protein family, is a four-member family of tyrosine kinase type I receptors that bind to ligands to form either homologous dimers or heterodimers that activate downstream Ras/Raf/MEK/ERK-MAPK or PI3K/AKT/mTOR signaling pathways, which eventually regulate tumor cell proliferation, invasion, and metastasis, including the suppression of tumor cell apoptosis [67]. In addition, extensive evidence has confirmed that various solid tumors overexpress EGFR, including GC [67, 68]. Therefore, these studies indicate that blocking the formation of EGFR dimers might be the starting point for suppressing tumor cell proliferation and for studying potential drug targets [68, 69]. In fact, according to the mechanism described above, clinical researchers have developed many related drugs, such as trastuzumab, pertuzumab, trastuzumab emtansine, and lapatinib [70]. Next, we explain the roles of these drugs in the treatment of GC. Trastuzumab, a recombinant humanized monoclonal antibody targeted to the extracellular domain IV of the human epidermal growth factor receptor 2 (HER2, also called neu gene, one of the oncogenes of GC), interferes with HER2 dimerization to directly initiate antibody-dependent cellular cytotoxicity by inhibiting cell proliferation, increase the role of intracellular phagocytic receptors, and even promote antiangiogenesis, thereby assuming an effective therapeutic role for patients with HER2-overexpressing advanced-stage GC [63, 66]. Pertuzumab, another human monoclonal antibody against the extracellular domain II of HER2 that also impedes its dimerization as well as ligand-activated signaling, was found to produce better results in GC patients with relatively low levels of HER2 expression [65]. Thus, because both trastuzumab and pertuzumab bind to different regions of the extracellular domain of HER2, their actions constitute a good complementary treatment for patients with HER2-positive advanced GC [71]. T-DM1, a novel antibody-drug conjugate of trastuzumab and maytansine 1 (a microtubule-inhibiting cytotoxicity-inducing drug), can disrupt the intracellular microtubule system and ultimately lead to cell cycle arrest and cell death in HER2-positive GC patients [72, 73]. Lapatinib, an oral tyrosine kinase inhibitor (TKI) that has a dual reversible inhibitory effect on EGFR and HER2, can suppress the activation of these kinases by binding to the intracellular ATP site and finally cause decreased cell proliferation and increased apoptosis in GC patients [70, 73]. Furthermore, several clinical studies have reported that lapatinib combined with chemotherapy drugs can provide a better curative effect for HER2-positive advanced-stage GC patients [65, 74]. Hence, all the final mechanisms involved in the treatment of GC by EGFR family-targeting agents are able to inhibit the proliferation of GC cells by suppressing the activation of the EGFR signaling pathway.

#### 2.1.2. Antiangiogenesis

Generally, during the early stage, many tumors primarily rely on the penetration of tissue fluids to maintain tumor growth [34]. However, when the tumor cells quickly grow into the surrounding tissue such that the penetration of tissue fluid cannot be used for their growth, the tumor cells induce the expression of epidermal growth factor (EGF) and fibroblast growth factor (FGF) in the blood vessels of the body to promote neovascularization, which provides additional nutrients for the proliferating tumor cells [13]. Therefore, VEGF and FGF play an extremely important role in tumor angiogenesis, which is one of the main causes of tumor growth and metastasis [75]. First, VEGF, an endothelial cell-specific mitogen and a mediator of vascular permeability, can selectively bind to its receptor (VEGFR) and trigger receptor dimerization and activation of downstream pathways, which eventually promotes vascular endothelial cell proliferation, differentiation, and tumor cell infiltration [76]. Moreover, some laboratory studies have demonstrated that the expression of VEGF is positively correlated with vascular proliferation and development of GC, and in addition, highly expressed VEGF can significantly reduce the survival rate of GC patients [77]. Therefore, these results suggest that blocking the VEGF-VEGFR signaling pathway might obstruct the proliferation of GC tissue and inhibit tumor growth. In the clinic, there have been some therapeutic drugs developed that aim to inhibit VEGF or VEGFR, such as bevacizumab, ramucirumab, sorafenib, and sunitinib [66]. Therefore, we elaborate on the effect of these drugs on GC therapy. Bevacizumab, a recombinant, humanized version of a murine anti-VEGF type A (VEGF-A) monoclonal antibody, was used in combination with chemotherapy (e.g., cisplatin, capecitabine, or fluorouracil) to treat patients with advanced GC in the AVAGAST phase III randomized trial by accelerating antiangiogenesis [63]. Ramucirumab, a novel fully human IgG1 monoclonal antibody targeted to VEGFR-2, was discovered to have significant antitumor activity and antiangiogenic effects as a single agent or in combination with other therapeutics in patients with advanced GC, which was verified by two placebo-controlled, double-blind phase III studies (REGARD trial and RAINBOW trial) [78]. Sorafenib, an oral small-molecule TKI with anti-VEGFR-2, anti-VEGFR-3, anti-PDGFR-b, anti-b-Raf, anti-c-Kit, or anti-Flt-3 activity, can directly affect tumor spread and inhibit angiogenesis [66, 73]. Sunitinib, similar to sorafenib, is another oral small-molecule TKI against VEGFR-1, VEGFR-2, VEGFR-3, PDGFR-a/b, Flt-3, c-Kit, and c-RET that exhibits only modest activity in the treatment of advanced-stage GC patients [65, 70]. Hence, these drugs collectively validate the supposition that the inhibition of the VEGF-VEGFR signaling pathway is an important therapeutic modality in advanced GC for use in developing antiangiogenic strategies.

### 2.2. Immunotherapy

Although the molecular targeted therapeutic drugs described above have been approved and used for the treatment of advanced GC, molecular targeted therapies for GC are still lagging behind those observed in other common Western diseases, such as lung cancer, breast cancer, and intestinal cancer [63]. Moreover, the heterogeneity of GC is very high, there are few targets to select, and there are poor results from targeted drugs tested in phase II and III clinical studies, meaning that the development of new treatment methods is urgently needed [79, 80]. In the past two decades, researchers have tried to adopt the body's own immune function to fight tumors in a strategy called tumor immunotherapy [81]. The purpose of tumor immunotherapy is to achieve therapeutic effects by enhancing the body's own antitumor immune response or exogenously supplementing antitumor immunocompetent cells and drugs to overcome the limitations of traditional treatments and provide new solutions for the treatment of cancer [82]. Currently, immunotherapy methods for tumors consist of nonspecific immunostimulation, adoptive cell transfer therapies (ACTs), tumor vaccines, and immune checkpoint inhibitors (ICIs) [81, 82]. An immune checkpoint is a mechanism by which the immune system maintains balance. When the body is infected by a pathogen, the immune checkpoint can protect the tissue cells from attack and is also a mechanism for tumor immune escape. Hence, the use of immune checkpoint inhibitors (ICIs) has attracted great attention from researchers to develop drugs for treating tumors by precisely regulating T cell activation. Among them, the programmed cell death protein 1 (PD-1)/the PD-1 ligand (PD-L1) axis played an important role. The PD-1 molecule is expressed on the surface of activated T cells, and PD-L1 is expressed in tumor cells. Moreover, when activated T cells and tumor cells bind to each other through the PD-1/PD-L1 axis, the functions of activated T cells were inhibited and finally resulted in tumor immune escape. Hence, targeted blocking of ICIs with monoclonal antibodies can effectively activate T cells and kill tumor cells. As is well known, the T cell activation needs 3 signals: (i) the interaction between the T cell receptor (TCR) and the major histocompatibility complex (MHC)/peptide; (ii) a costimulatory signal defined as the interaction between CD28 molecules expressed on T lymphocytes and CD80/CD86 (B7 molecules) expressed on antigen-presenting cells (APC); and (iii) the IL-2/IL-2 receptor signaling pathway. These 3 signals lead to lymphocyte cycle progression, survival, and differentiation. Therefore, any factor affecting these three signals may directly affect the activation of T cells. In the original manuscript, we described that “immune checkpoint inhibitors (ICIs) enhance the adhesive ability to antigen-presenting cells and cytotoxic T cells,” which referred to the above described (ii) signal. Although there were no clinical experiments that demonstrated that ICIs could directly enhance the contact between antigen-presenting cells and cytotoxic T cells, this is a new direction for cancer drug development based on the fact that the checkpoint pathways are regulated by ligand/receptor interactions.

Next, we briefly introduce the applications of these immunotherapies in the treatment of GC. Nonspecific immunostimulation therapy, such as streptococcal preparation (OK-432) and lentinan, enhances the immune effect by promoting the activity of T cells and NKs and the release of various cytokines, which can produce anticancer immunity at the initial stage of tumor formation [83]. ACTs represent a novel therapeutic method that uses normal immune effector cells with antitumor activity (e.g., dendritic cells (DCs), natural killer cells (NKs), lymphokine-activated killer cells (LAKs), tumor-infiltrating lymphocytes (TIL), cytokine-induced killer cells (CIK), and chimeric antigen receptor T cells (CAR-T)) that were first extracted from patients, expanded or cultured *in vitro*, and finally administered into the tumor patients to kill the tumor cells [84]. A clinical trial has uncovered that ACT with TIL plus chemotherapy leads to a higher overall survival rate than chemotherapy alone in advanced GC patients, which implies that ACT might improve the efficacy of therapeutic effects through different synergistic mechanisms than those of chemotherapy [85]. Tumor vaccines take advantage of tumor-associated antigens (i.e., antigens expressed on tumor cells) that may be recognized as foreign to activate and expand tumor-specific effector T cells, which further enhance preexisting immunity and elicit a more robust antitumor immune response to eliminate tumor cells [86]. For example, a HER2/DC vaccine consisting of DCs and HER2/neu peptide was confirmed to have a strong therapeutic action in HER2-positive GC patients [87]. ICIs are mainly used to suppress immune checkpoints, which eventually results in promoting the killing effect of autoimmune cells on tumor cells [88]. Currently, there are two important targets of ICIs: inhibitors of cytotoxic T lymphocyte antigen 4 (CTLA-4) and inhibitors of programmed cell death protein 1 (PD-1) and its ligands (PD-L1) [89, 90]. Several studies have shown a PD-1/PD-L1 axis overexpression trend in GC patients; thus, blocking the PD-1/PD-L1 axis might facilitate T cell antitumor activity against the tumor cells of GC patients [90]. Moreover, as is well known, T cell activation requires 3 signals: (i) the interaction between the T cell receptor (TCR) and the major histocompatibility complex (MHC)/peptide; (ii) a costimulatory signal defined as the interaction between CD28 molecules expressed on T lymphocytes and CD80/CD86 (B7 molecules) expressed on antigen-presenting cells (APC); and (iii) the IL-2/IL-2 receptor signaling pathway. These 3 signals lead to lymphocyte cycle progression, survival, and differentiation. Therefore, any factor affecting these three signals may directly affect the activation of T cells; for instance, ICIs enhance the adhesive ability of antigen-presenting cells to cytotoxic T cells, which might be a new direction for cancer drug development based on the fact that the checkpoint pathways are regulated by ligand/receptor interactions. Collectively, although the immunotherapies of GC are still in their infancy, immunotherapies have constituted a new direction in the field of GC with the continuous growth in the understanding of the interaction among the tumor, the tumor microenvironment, and the host immune system.

### 2.3. Small Molecular Therapy

Ever since the discovery of lncRNAs, accumulating evidence has provided a new horizon for understanding the orchestrated regulation of several genes involved in carcinogenesis and in malignant phenotype maintenance [51]. Therefore, lncRNAs utilized as biomarkers for assessing the prognosis of cancer patients or as target molecules for the development of emerging specifically targeted drugs have been widely pursued [48]. Presently, many studies focus on the interactions between lncRNAs and GC resistance, and most of them mainly address multidrug resistance, especially resistance to doxorubicin, cisplatin, and fluorouracil [91]. It has been reported in many studies that lncRNAs induce drug resistance by regulating DNA damage and the cell cycle, thereby affecting drug transport systems, interfering with drug metabolism, disrupting tumor cell apoptosis, mediating the EMT process, and so on [92]. For example, ATP-binding cassette (ABC) superfamily members are important drug transporters that affect the sensitivity of chemotherapeutic drugs, and their effects on MDR are particularly prominent [93]. However, it was discovered that dysregulated lncRNAs could participate in the regulation of tumor chemoresistance by mediating the expression of ABC superfamily proteins during the progression of GC [92]. Moreover, some studies have clearly revealed that the lncRNA ANRIL is significantly upregulated in GC patients who are administered cisplatin and 5-fluorouracil treatment and who develop drug resistance, and inhibition of lncRNA ANRIL can reverse the resistance to cisplatin and 5-fluorouracil by reducing the expression of MDR-associated proteins, such as multidrug resistance 1 (MDR1) and mitochondrial 37S ribosomal protein 1 (MRP1) [94]. Additionally, EMT refers to cells losing their epithelial properties and obtaining interstitial properties, which gives them enhanced cell motility, and eventually, they break through the intercellular adhesions to advance cellular metastasis. Studies have confirmed that the increased ability of cell motility could help cells escape drug stimulation, resulting in drug resistance [34]. Multiple signaling pathways in tumor cells are involved in the development of EMT, including Wnt/*β*-catenin signaling, TGF-*β* signaling, and AKT/mTOR signaling [13, 95]. Recent documentation on a variety of lncRNAs implicates them in the regulation of EMT-related signaling pathways that may affect the formation of tumor cell resistance [96]; for example, lncRNA HOTAIR can activate the PI3K/AKT/MRP1 pathway to increase the resistance of GC cells to cisplatin [97]. Furthermore, uncontrolled apoptosis is another major factor in the development of drug resistance, mainly because some tumor chemotherapy drugs could inhibit the growth of tumor cells by inducing apoptosis [98]. It was reported that lncRNA UCA1 regulated the resistance of GC to doxorubicin by affecting the apoptotic pathway; specifically, silencing lncRNA UCA1 expression could promote the apoptosis of GC cells induced by doxorubicin by upregulating the expression of the PAPP protein and inhibiting the expression of the antiapoptotic protein Bcl-2 [99]. In fact, there have been many other lncRNAs verified as involved in the drug resistance observed in GC therapy, the details of which are shown in Table 2.

## 3. Conclusion

China is a country with a high GC morbidity rate, which accounts for one-half of the new cases worldwide, and most GC patients are diagnosed at an advanced stage after they have lost the best chance of successful surgical treatment, and their prognosis is extremely poor [1, 2]. With the popularization and application of standardized treatment of tumors, early- and middle-stage GC patients have received great attention, and surgery remains the only curative therapy for these patients [62]. However, although the treatment methods and therapeutic effects have been significantly improved in recent years, there are still no effective treatments for advanced-stage GC patients [15, 61]. In the past, chemotherapy was the most common treatment for advanced-stage GC patients, but due to the chemotherapy drugs having extensive side effects in GC patients and the easily produced drug resistance, many emerging treatments are being developed rapidly, including those based on molecular targeted therapy, immunotherapy, and small molecular therapy [62, 79]. In summary, from the above discussion, we know the following. (1) The molecular targeted therapy treatment method is primarily based on the pathogenic mechanism of GC, but in recent years, most of the studies have failed, which has made scholars realize the importance of finding related molecular markers and adapting them to the selected population, but only two drugs (i.e., trastuzumab and ramucirumab) have been approved for the market [21, 66]. (2) Immunotherapy, as a new type of anticancer treatment, can be used to detect and eliminate malignant tumors by activating the body's own immune system, which has very broad treatment prospects. Nevertheless, because the microenvironment of the tumor is rather complex, the microenvironments in the patients who undergo multiple chemotherapies may change, and then, the immune function of the patients also decreases, creating major challenges for immunotherapy in the future [81, 82]. (3) Small molecular therapy, especially that based on lncRNAs, is expected to become a more reasonable and comprehensive treatment plan because of the crucial roles of lncRNAs during the occurrence, development, and progression of GC. Based on the various shortcomings of the treatment methods described above, including the drug resistance to chemotherapy, the clinical trial failure of molecular targeted therapy, and the individual differences in immunotherapy, some researchers were surprised to find that treatments specifically targeting lncRNAs might resolve these above issues [32]. Thus, the effects of lncRNAs in GC are gradually being elucidated, their clinical application value will also need to be gradually tested, and this process may create new possibilities for solving the problem of chemotherapy resistance, precision-targeted therapy, and individualized treatment plans in GC patients [92]. Nonetheless, it is undeniable that there are still many challenges in the application of lncRNAs in the treatment of GC. For instance, advancing the clinical transformation of lncRNA-targeted therapy is very difficult, which means that successful lncRNAs in cell and animal models do not necessarily translate in the clinic. Collectively, although there are still no effective measures for the treatment of advanced GC, these emerging treatment programs provide theoretical support for creating precise treatments. It is believed that there will definitely be a breakthrough in the treatment of GC in the future.

## Figures and Tables

**Figure 1:** The classification and biological roles of lncRNAs.

**Figure 2:** lncRNAs associated with drug resistance in GC.

**Table 1:** Expression of lncRNAs associated with human GC.

lncRNAs	Location	Expression	Samples	Function in tumorigenesis	References
AK058003	10q22	Upregulated	GC tissues, SGC7901 cell, and MKN45 cell	Relates to cell growth, invasion, metastasis, lymph node metastasis, and clinical stages	[100]
ANRIL (antisense noncoding RNA in the INK4 locus)	9p21.3	Upregulated	GC tissues	Promotes tumor growth and metastasis	[101]
ATB (activated by TGF-*β*)	Chromosome 14	Upregulated	GC tissues, MGC803 cell, MKN45 cell, BGC823 cell, MKN28 cell, and SGC7901 cell	Associates with EMT, migration, and vascular invasion	[102]
BANCR (BRAF activated noncoding RNA)	Chromosome 9	Upregulated	GC tissues, MGC803 cell, and BGC823 cell	Biomarker in the clinical stage, tumor depth, lymph node metastasis, and distant metastasis	[103]
CCAT1 (colon cancer-associated transcript 1)	8q24.21	Upregulated	GC tissues	Oncogene	([104]; [105])
FENDRR (FOXF1 adjacent noncoding developmental regulatory RNA)	16q24.1	Downregulated	GC tissues, MGC803 cell, BGC823 cell, MKN28 cell, MKN45 cell, and SGC7901 cell	Inhibits invasion and migration	[106]
FER1L4 (Fer-1 like family member 4)	20q11.22	Downregulated	GC tissues	A potential biomarker in the diagnosis of GC	[107]
GACAT1/2 (gastric cancer-associated transcript 1/2)	2q12.3/18p11	Downregulated	GC tissues, BGC823 cell, MGC803 cell, SGC7901 cell, and HGC2 cell	A potential biomarker in the diagnosis of GC	[108]
GAPLINC (gastric adenocarcinoma associated, positive CD44 regulator, long intergenic noncoding RNA)	18p11	Downregulated	GC tissues, KATO III cell, HGC27 cell, and SNU1 cell	Poor survival and prognosis marker	[109]
GAS5 (growth arrest-specific 5)	1q25.1	Downregulated	GC tissues and cell lines	Suppresses cell proliferation	([110]; [111])
GHET1 (gastric carcinoma proliferation enhancing transcript 1)	7q36.1	Upregulated	GC tissues and cell lines	Promotes cell proliferation	[63]
H19 (human homologue 19)	11p15.5	Upregulated	GC tissues, BGC823 cell, MGC803 cell, and MKN45 cell	Promotes cell growth, proliferation, invasion, EMT	([112]; [113])
HIF1A-AS2 (HIF1A antisense RNA 2)	Chromosome 14	Upregulated	GC tissues and cell lines	Diagnostic and prognostic marker	[114]
HOTAIR (HOX antisense intergenic RNA)	12q13.13	Upregulated	GC tissues, AGS cell, SGC7901 cell, MGC803 cell, and BGC823 cell	Function as ceRNA to regulate HER2 by sponging miR-331-3p or STAT3/cyclin D1 by sponging miR-454-3p; promote EMT and invasiveness	([115]; [116])
HOXA-AS2 (HOXA cluster antisense RNA2)	7p15.2	Upregulated	GC tissues, BGC823 cell, SGC7901 cell, AGS cell	Associates with tumor size and clinical stage	[117]
HULC (highly upregulated in liver cancer)	6p24.3	Upregulated	GC tissues, SGC7901 cell, MKN28 cell, MKN45 cell, AGS cell, and BGC823 cell	Promotes proliferation and invasion and inhibits apoptosis	[118]
LINC00152 (also termed CYTOR, cytoskeleton regulator RNA)	Chromosome 2	Upregulated	GC tissues, BGC823 cell, MGC803 cell, and SGC7901 cell	Predicts GC prognosis	[119]
LINC00982 (also named PRDM16-DT PRDM16 divergent transcript)	Chromosome 1	Downregulated	GC tissues and cell lines	Prognostic marker	[120]
LSINCT (the lncRNA long stress-induced noncoding transcript 5)	5p15.33	Upregulated	GC tissues	Associates with TNM stage, tumor size, and depth of invasion	[121]
MALAT1 (metastasis-associated lung adenocarcinoma transcript 1)	11q13.1	Upregulated	GC tissues, BGC823 cell, SGC7901 cell, and HGC27 cell	Promotes cell proliferation and invasion	([122]; [123])
MEG3 (maternally expressed gene 3)	14q32.2	Downregulated	GC tissues, SGC7901 cell, AGS cell, MGC803 cell, MKN45 cell, and MKN28 cell	Suppresses cell proliferation and metastasis	([124]; [53])
MRUL (MDR-related and upregulated lncRNA)	400 kb downstream of ABCB1	Upregulated	GC tissues	Indicates a poor prognosis for GC patients	[125]
PVT1 (Pvt1 oncogene)	8q24	Upregulated	GC cell lines	A new biomarker for GC and indicate lymph node invasion	[126]
SNHG5 (small nucleolar RNA host gene 5)	6q14.3	Downregulated	GC tissues, SGC7901 cell, and MGC803 cell	Suppresses cell proliferation and metastasis	[127]
Sox2ot (SOX2 overlapping transcript)	Chromosome 3	Upregulated	GC tissues and cell lines	Promotes cell growth and motility	[128]
SUMO1P3 (small ubiquitin-like modifier 1 pseudogene 3)	20q11.22	Upregulated	GC tissues	A potential biomarker in the diagnosis of GC	[129]
TUSC7 (tumor suppressor candidate 7)	3q13.31	Downregulated	GC tissues, AGS cell, and MKN45 cell	Hinders tumor cell growth	[130]
UBC1 (upregulated in bladder cancer 1)	1q32.1	Upregulated	GC tissues	Associates with lymph node metastasis, tumor size, TNM stage, and poorer prognosis in GC	[131]
UCA1 (urothelial carcinoma associated 1)	19p13.12	Upregulated	GC tissues	Associates with tumor size, differentiation, invasion depth, and TNM stages	[132]

**Table 2:** lncRNAs associated with drug resistance in the treatment of GC.

lncRNAs	Location	Expression	Drugs	Mechanism	References
AK022798	—	Upregulated	Cisplatin	Notch 1 can promote the lncRNA AK022798 expression and result in the formation of SGC7901/cisplatin and BGC823/cisplatin cells.	[133]
BCAR4 (breast cancer anti-estrogen resistance 4)	16p13.13	Upregulated	Cisplatin	Overexpression of BCAR4 in SGC7901 cells increased resistance to cisplatin, while reduced BCAR4 expression increased the sensitivity of SGC7901/cisplatin cells to cisplatin.	[134]
CASC2 (cancer susceptibility 2)	10q26.11	Downregulated	Cisplatin	CASC2 overexpression overcame cisplatin resistance in gastric cancer by sponging miR-19a.	[135]
CASC9 (cancer susceptibility 9)	8q21.13	Upregulated	Paclitaxel, adriamycin	CASC9 knockdown restored chemosensitivity to paclitaxel and adriamycin by decreasing the expression of MDR1protein.	[136]
GHET1 (gastric carcinoma proliferation enhancing transcript 1)	7q36.1	Upregulated	Cisplatin	Highly expressing GHET1 promoted the development of MDR, which was related to the Bax, Bcl-2, MDR1, and MRP1 gene expression in gastric cancer cells.	[137]
LEIGC	—	Downregulated	5-Fluorouracil	Overexpression of LEIGC suppressed tumor growth and cell proliferation and enhanced the sensitivity of gastric cancer cells to 5-fluorouracil, whereas knockdown of LEIGC showed the opposite effect.	[138]
MALAT1 (metastasis-associated lung adenocarcinoma transcript 1)	11q13.1	Upregulated	Vincristine, cisplatin	MALAT1 acts as a competing endogenous RNA for miR-23b-3p and attenuates the inhibitory effect of miR-23b-3p on ATG12, leading to chemo-induced autophagy and chemoresistance in GC cells.	[139]
MRUL (also named DMTF1, cyclin D-binding myb-like transcription factor 1)	7q21.12	Upregulated	MDR	MRUL depletion reduced ABCB1 mRNA levels in a dose- and time-dependent manner, and ABCB1 was responsible for drug transporters.	[140]
PTV1 (polytropic virus 1)	—	Upregulated	Cisplatin	Overexpression of lncRNA PVT1 in gastric carcinoma promotes the development of MDR.	[141]
XLOC_006753	—	Upregulated	MDR	High expression of XLOC_006753 promoted the development of MDR, which was activated by the PI3K/AKT/mTOR pathway in GC cells.	[142]
ZFAS (zinc finger antisense)	Chromosome 8	Upregulated	Cisplatin, paclitaxel	The silencing of ZFAS1 inhibited the growth, proliferation, cell cycle progress, migration, invasion, EMT, and chemotherapeutic tolerance by blocking the Wnt/*β*-catenin signaling in gastric cancer cells.	[143]

## Data Availability

The datasets during the current study are available from the corresponding author on reasonable request.

## Abbreviations

GC: Gastric cancer
lncRNAs: Long noncoding RNAs
ORF: Open reading frame
spRNAP IV: Single-polypeptide nuclear RNA polymerase IV
TFs: Transcription factors
ncRNAs: Noncoding RNAs
miRNAs: MicroRNAs
siRNAs: Small interfering RNAs
piRNAs: Piwi-interacting RNAs
rRNAs: Ribosomal RNAs
tRNAs: Transfer RNAs
snRNAs: Small nuclear RNAs
snoRNAs: Small nucleolar RNAs
EMT: Epithelial-mesenchymal transition
FoxQ1: Forkhead box Q1
CAB39: Calcium-binding protein 39
lncRNA SNHG7: Long noncoding small nucleolar RNA host gene 7
lncRNA MEG3: Long noncoding maternally expressed gene 3
ceRNAs: Competing endogenous RNAs
ZEB2-AS1: Zinc finger E-box-binding homeobox 2 antisense RNA 1
ANRIL: Antisense noncoding RNA in the INK4 locus
CCAT1: Colon cancer-associated transcript 1
FENDRR: FOXF1 adjacent noncoding developmental regulatory RNA
FER1L4: Fer-1 like family member 4
GACAT1/2: Gastric cancer-associated transcript 1/2
GAPLINC: Gastric adenocarcinoma associated, positive CD44 regulator, long intergenic noncoding RNA
GAS5: Growth arrest-specific 5
GHET1: Gastric carcinoma proliferation enhancing transcript 1
H19: Human homologue 19
HIF1A-AS2: HIF1A antisense RNA 2
HOTAIR: HOX antisense intergenic RNA
LSINCT: The lncRNA long stress-induced noncoding transcript 5
MALAT1: Metastasis-associated lung adenocarcinoma transcript 1
MRUL: MDR-related and upregulated lncRNA
SNHG5: Small nucleolar RNA host gene 5
SUMO1P3: Small ubiquitin-like modifier 1 pseudogene 3
UBC1: Upregulated in bladder cancer 1
TUSC7: Tumor suppressor candidate 7
UCA1: Urothelial carcinoma associated 1
HER2: Human epidermal growth factor receptor 2
EGF: Epidermal growth factor
FGF: Fibroblast growth factor
ACTs: Adoptive cell transfer therapies
ICIs: Immune checkpoint inhibitors
DCs: Dendritic cells
NKs: Natural killer cells
LAKs: Lymphokine-activated killer cells
TIL: Tumor-infiltrating lymphocytes
CIK: Cytokine-induced killer cells
CAR-T: Chimeric antigen receptor T cells
CLTA-4: Cytotoxic T lymphocyte antigen 4
ABC: ATP-binding cassette
MDR1: Multidrug resistance 1
MRP1: Mitochondrial 37S ribosomal protein 1
CASC2: Cancer susceptibility 2
CASC9: Cancer susceptibility 9
PTV1: Polytropic virus 1
ZFAS: Zinc finger antisense.
